# The effects of short interventions of focused-attention vs. self-compassion mindfulness meditation on undergraduate students: Evidence from self-report, classroom performance, and ERPs

**DOI:** 10.1371/journal.pone.0278826

**Published:** 2023-01-20

**Authors:** Aminda J. O’Hare, Zachary T. Gemelli

**Affiliations:** 1 Department of Psychological Science, Weber State University, Ogden, Utah, United States of America; 2 Department of Psychology, University of Massachusetts Dartmouth, Dartmouth, Massachusetts, United States of America; Sapienza University of Rome, ITALY

## Abstract

Mindfulness-based stress reduction (MBSR) training has been shown to improve cognitive processing, wellbeing, and academic performance. However, mindfulness interventions that are integrated into non-mindfulness related courses have not been well-investigated. Further, the unique effects of different aspects of MBSR training are not as well understood. This paper examines the effects that are uniquely associated with focused-attention versus self-compassion mindfulness practices utilizing a multi-method approach. Event-related potentials (ERPs) were recorded during an Emotional Flanker task, and self-report measures of wellbeing and measures of classroom performance were collected before and after training. Participants were students in two sections of the same undergraduate course and either completed 10 weeks of focused-attention practice or self-compassion practice that was built into their class sessions. Students in the focused-attention group (mean age = 22.08) had reduced interference effects on their reaction times following the training. Students in the self-compassion group (mean age = 23.91) showed altered processing of conflict on negative trials via the N2 and P3 ERP amplitudes after the training. This group also reported significant improvements in wellbeing and performed significantly better on more class tests compared to the focused-attention group. These data support the effectiveness of incorporating brief, simplified mindfulness practices in any classroom as an intervention to improve attention, wellbeing and classroom performance.

## Introduction

The benefits of mindfulness practices for wellbeing in educational settings have been established. While most research in this area has focused on primary and secondary schools [1, 2], the literature on the benefits of mindfulness practices in higher education is also growing [3]. How improved wellbeing impacts academic performance has not been as well explored, the interventions used for these studies typically employ time-intensive practices or mindfulness-dedicated courses, and a variety of mindfulness techniques are typically used in combination for the interventions. In order for mindfulness practices to be more widely incorporated into higher education classrooms, evidence that supports brief, simple interventions is needed. Further, better understanding the unique contributions of different types of mindfulness techniques can inform instructors on which practices may be best for their students, their students’ learning, and/or their students’ wellbeing.

Mindfulness, as defined by Jon Kabat-Zinn, is the “awareness that emerges through paying attention on purpose, in the present moment, and nonjudgmentally to the unfolding of experience moment-by-moment” [4, p. 145]. Specifically, it is the intentional regulation of attention with an open and non-judgmental attitude [5, 6]. Mindfulness improves self-regulation and self-management, emotional and cognitive flexibility, and clarification of values [6]. A meta-meta analysis found mindfulness based interventions (MBIs) to benefit those with psychiatric disorders and alleviate both psychiatric and physiological symptoms of their diagnosed disorder(s) [7].

The most common type of MBI found in the literature is Mindfulness-Based Stress Reduction (MBSR), an intervention developed by Kabat-Zinn [8]. This intervention lasts 8 weeks and includes several different mindfulness techniques, such as body scans, mindful breathing, mindful walking, mindful eating, hatha yoga, and loving-kindness or metta meditation. Participants meet as a group for 2–4 hours weekly to learn new techniques and are asked to practice 15–45 minutes daily on their own. The intervention ends with a 4 hour half day silent retreat. Most research on the benefits of mindfulness practices includes various forms of these practices from MBSR in the study interventions or rely on correlational approaches with expert meditators [9], so the unique effects of different types of mindfulness practices are not as well understood. Those that have compared different mindfulness techniques have found unique mechanisms to similar outcomes; however these studies are not conducted in educational contexts [10–12].

Two types of mindfulness practices that have been examined individually are 1) loving-kindness or metta practices and 2) breath-focused attention practices. Loving-kindness or metta mindfulness practices are typically used to enhance an individual’s capacity for compassion [13]. In MBSR interventions, participants progressively practice generating compassion towards loved ones, themselves, individuals who are causing conflict, and all beings [8]. Specifically, self-compassion mindfulness, when compassion is generated towards oneself through the focus on a basic mantra of compassion directed toward oneself, has been shown to improve states of wellbeing [14].

A meta-analysis observed that various forms of kindness-based meditation interventions, including compassion practices, were moderately effective in decreasing self-reported depression and increasing mindfulness, compassion, and self-compassion compared to passive controls [15]. This same review also observed that positive emotions were increased through kindness-based meditations compared to practicing progressive relaxation. Supporting these findings, Haukaas and colleagues observed that both mindful self-compassion and attention training interventions (3 weekly sessions for 45 minutes) reduced depression and anxiety, while significantly increasing mindfulness, and self-compassion post-intervention [16]. Finally, Klimecki and colleagues found individuals to report improved positive affect and reduced negative affect following compassion training when compared to empathy training [13].

Mindfulness practices have also been found to impact attention. One particular aspect of mindfulness, focused-attention (FA) mindfulness, has been shown to enhance attention processes. In FA mindfulness, individuals direct their attention to a single sensory input, commonly the sensation of the breath [8]. One study comparing FA mindfulness to socio-cognitive and socio-affective interventions, observed an enhancement of attentional control specific to the FA group post-intervention [17]. The intervention consisted of 13 weeks of daily practice in addition to a 2-hour weekly group session and a one-time 3-day retreat. Supporting this effect, a systematic review observed that mindful breathing (FA) reduced interference on a Stroop task, indicating improvements in attentional control [18]. FA mindfulness has also been found to increase post-intervention self-reported breath focus and attention shift abilities [19].

In educational settings, MBIs have been found to enhance both student wellbeing and academic performance. This research started in primary and secondary school interventions [1, 2], but it has been expanding into exploring the effects of MBIs in higher education [3]. For example, Lin and Mai studied the effects of three months of mindfulness meditation for 10–20 minutes per week in college students compared to controls [20]. Both groups, in the same college course, took in-class quizzes after each class (short-term) and two summative assessments after multiple classes (long-term). At the beginning of each class, the control group would review notes for the first 10–20 minutes of each class, while the experimental group would participate in mindfulness for the first 10–20 minutes of each class. As predicted, the mindfulness group had better short-term academic performance, however, both groups had similar long-term academic performance. Interestingly, within the mindfulness group those with higher meditation depth (as measured by self-report) experienced higher short-term performance compared to those with lower meditation depth. The impact of mindfulness meditation on students’ wellbeing was not assessed in this study.

Another study by Franco and colleagues also observed increased academic performance in high school students by implementing an MBI [21]. The students who participated in a 10-week mindfulness intervention (30 minutes of practice per week) significantly improved in academic performance (subject grades) and decreased in state and trait anxiety compared to controls. Following these results, Beauchemin and colleagues observed that high school students with learning disabilities who completed a five-week MBI also experienced attenuated state and trait anxiety, as well as heightened social skills with others, and enhanced academic performance compared to pre-intervention [22]. The intervention started with a single 45-minute practice, followed by 5 to 10 minutes of practice at the beginning of each class for 5 weeks. These studies indicate that incorporating mindfulness practices into classroom environments can have benefits for classroom performance as well as student wellbeing, but they do not indicate if a compassion-based or attention-based intervention has greater effects.

What can inform the type of MBI most appropriate for different educational settings is a better understanding of the mechanisms that drive the effects of mindfulness practices on wellbeing and academic performance. Electrophysiology is a methodology of cognitive neuroscience that can provide insight into these mechanisms. Event-related potentials (ERPs) are neural components derived from electroencephalography (EEG) data that are sensitive to changes in information processing with millisecond accuracy. ERP studies have been used to study both the wellbeing and attention effects of mindfulness.

For example, one ERP study showed that mindfulness meditation attenuated the impact of negative stimuli on the LPP component, which is a neural index of sustained, motivated attention to emotionally salient stimuli [23]. Sanger and colleagues found an 8-week mindfulness training group (8 weekly sessions of 50 minutes) to have significant increases in self-reported wellbeing and fewer doctor visits for mental health support compared to controls [24]. These effects were accompanied by the mindfulness group having a sustained P3b component to target stimuli in an emotional oddball task compared to a control group. The P3b component is a neural index of selective attention to relevant stimuli [25].

Numerous ERP studies have evidenced attentional control enhancements from mindfulness meditation through improvements on tasks that depend on attentional control [25–28]. The most commonly impacted ERP components in this research are the N2 and the P3. The N2 is a neural index of conflict monitoring that signifies the inhibition of bottom-up processes (i.e., automatic response processes) through the use of top-down mechanisms [29–33]. For example, in tasks engaging cognitive control, such as the Flanker task, larger N2 responses are elicited by incongruent stimuli compared to congruent [34], and reductions in the N2 response are associated with improvements in performance [35]. The P3 is a neural index of selective attention, stimulus evaluation, context updating, and the facilitation of memory processing [9, 25, 32, 36, 37]. For example, emotional stimuli evoke larger P3 responses than non-emotional due to their engagement of attention and working memory [38]. Reductions in P3 responses to distracting stimuli indicate that selective attention is being less engaged by these stimuli.

Atchley and colleagues observed that expert meditators could modulate their N2 and P3 responses depending upon the focus of attention [9]. In an auditory oddball task, meditators had a significant increase in N2 and P3 amplitudes when attending to target stimuli compared to controls. In a subsequent breath counting task, when instructed to ignore the same auditory stimuli, meditators had an attenuation of the N2 and P3 amplitudes. These data indicate that meditators were better able to control attention toward target stimuli and away from distracting stimuli when that was their intention, and that the N2 and P3 components were modulated by this control of attention. In this study, groups were defined as being meditators (novice or expert) or non-meditators (naive/controls) according to their self-reported meditation experience.

Another study by Quaglia and colleagues unilized a 4-week FA mindfulness intervention that required a 20-minute practice once per week [33]. Post-intervention, FA mindfulness facilitated better conflict monitoring on an emotional go/no-go task compared to active controls. This was indexed by shorter response time and accuracy, as well as an increase in N2 ERP amplitude compared to active controls. Finally, Moore and colleagues employed 16 weeks of FA mindfulness practice following a 2 hour training session and instructions to practice at least 10 minutes per day for 5 days a week, and found ERP indices of improved attentional control on a Stroop task in participants [39].

### The present study

The present study aims to further examine the unique effects of self-compassion (SC) and focused-attention (FA) mindfulness practices in higher education settings using a multi-method approach by assessing students’ self-report measures of wellbeing, classroom performance, and ERPs during a cognitive task with emotional distraction. We provide a novel approach by combining both applied educational assessments and experimental laboratory assessments of two different MBIs. Participants were students in two sections of the same undergraduate course who either completed a semester of FA practice or a semester of SC practice. Students’ grades on course tests were compared, and they completed self-report measures of wellbeing before and after the intervention. An emotional variant of a traditional cognitive paradigm for examining attentional control, the Eriksen Flanker Task [40], was created by priming flanker stimuli with emotion words to examine the cognitive mechanisms impacted by the MBIs. Flanker stimuli consist of a center arrowhead (<) flanked by other arrowheads on either side (e.g., <<<<<). Participants are tasked with indicating the direction the center arrowhead is pointing. This task can be used to assess attentional control by comparing incongruent (e.g., <<><<) to congruent (e.g., <<<<<) trials, as well as emotional distraction by comparing negative to neutral trials.

While the literature supports that most mindfulness interventions improve classroom performance, compassion practices also significantly increase wellbeing. As such, we predicted that the SC group would perform significantly better on course tests than the FA group, and the SC group would self-report greater wellbeing than the FA group. In this way, the SC practice serves as a “double-edged sword” by helping to improve attention as well as reducing emotional distraction, such as test anxiety, to improve test performance.

For the Emotional Flanker task, we predicted that negative primes would evoke larger ERP responses to Flanker stimuli due to engaging more attention and distraction on those trials. We predicted that participants completing the FA practice would show greater improvements in attentional control, as indicated by reduced interference on the Flanker task on reaction times and decreased N2 and P3 ERP amplitudes on incongruent trials. For participants completing the SC practice, we predicted greater improvements in attentional control specifically when negative emotion was present, as indicated by reduced interference on negative flanker trials on reaction times and decreased N2 and P3 ERP amplitudes.

## Method

### Participants

Participants were recruited from two undergraduate classes in Biopsychology at a university in the New England region of the United States. This study was approved by the University of Massachusetts Dartmouth Internal Review Board. Written, informed consent was obtained from all participants. One class was randomly assigned to engage in focused-attention mindfulness (FA Group), and the other class was assigned to engage in self-compassion mindfulness (SC Group). These classes resulted in a possible participant pool of 37 for the focused-attention class and 35 for the self-compassion class. For participating in this study, individuals were awarded extra credit for completion on each aspect of participation. During the first three weeks of the semester (pre-training), students could elect to participate by 1) having their test grades analyzed, 2) completing the online self-report measures, and/or 3) coming to a lab to complete an emotional Flanker task while EEG data was recorded. Mindfulness training started in the classes during the fourth week of the semester and continued until week 13 (10 weeks total). During the last week and a half of the semester (post-training), participants from the pre-training data were asked to complete the online self-report measures and/or the lab task with EEG again. There was no exclusionary criteria for participating in this study; however some incomplete survey or noisy EEG data was removed after data collection. Participants were not screened for neurological and psychiatric comorbidities, and were not screened for prior mindfulness experience. The groups did not significantly differ on age (FA Group M age = 22.08 years, SD = 7.26; SC Group M age = 23.91, SD = 6.51) or gender (FA Group = 15.38% male, SC Group = 13.04% male) proportions. Four participants were removed due to being left-handed specifically in the EEG data. The sample sizes for participation in these different parts of the study can be found in Fig 1. For the FA Group, 31 participants completed the pre-intervention online self-report measures and 24 completed the post-intervention online self-report measures, while 23 completed the pre-intervention lab task and 15 completed the post-intervention lab task. For the SC Group, 24 participants completed the pre-intervention online self-report measures and 20 completed the post-intervention online self-report measures, while 24 completed the pre-intervention lab task and 16 completed the post-intervention lab task.

**Fig 1:** Consort flow diagram indicating inclusion and participation of participants at different stages of the study.

### Mindfulness practices

Both classes met twice a week on Tuesdays and Thursdays for 75 minute periods. Both classes were taught by the same instructor, and the content covered and the pace of content covered in each class was identical. The first five minutes of each class were used for the assigned mindfulness practice. The rest of the time was the Biopsychology course as usual. As such, each group practiced for 10 minutes per week. The course instructor also led the mindfulness practices. She completed three semesters of training in a clinical psychology doctoral practicum in MBSR group work and ran a faculty forum on incorporating mindfulness practices into higher education. The FA practice was reduced to breath-focused mindfulness meditation only. The SC practice was reduced to meditation focusing on phrases of self-compassion only. Participants were not asked to practice outside of class.

#### Focused-attention mindfulness meditation

Once class started, participants were asked to sit up straight with their eyes closed. They were instructed to bring their attention to the sensation generated by their breath and work on letting go of other thoughts or mind-wandering. Verbal cues were given intermittently throughout the practice to remind participants to stay present with the sensation of the breath. At the end of the five minutes, participants were asked to take a deep, focused breath together and open their eyes.

#### Self-compassion mindfulness meditation

Once class started, participants were asked to sit up straight with their eyes closed. They were instructed to bring their attention to specific phrases or “mantras” by saying them silently to themselves and work on letting go of other thoughts or mind-wandering. The phrases of self compassion were, “May I be happy,” “May I be calm,” and “May I be well”. Verbal cues were given intermittently throughout the practice to remind participants to stay present with the phrases of self-compassion. At the end of the five minutes, participants were asked to silently finish the phrase they were on and open their eyes.

### Materials

#### Course tests

There were four section tests for these courses. The tests were identical for each course. Testsconsisted of multiple choice questions, diagram labeling, and short answer questions relevant to the content of the most recent section of the course. Test 1 was given on week 3. The mindfulness practices started the class after Test 1 was administered. As such, Test 1 serves as a pre-mindfulness training assessment to compare academic performance between the two courses. Test 2 was given on week 6, Test 3 was given on week 9, and Test 4 was given on week 13. Classes met only once on weeks 10 and 12 due to university holidays.

#### EEG equipment and recording

We used BioSemi: ActiveTwo Ag/AgCl active electrodes to record EEG from 64 channels that we positioned according to the international 10–20 system [41]. Signa gel, a saline-based gel, was applied to each of the 64 channels to conduct signals. External electrodes were also applied on both mastoids and below the right eye to record vertical eye movements (VEOG) and to the right of the same eye to record horizontal eye movements (HEOG). All impedances were set below 50 kΩ, the signal was preamplified at the electrode with a gain of 16x, and the EEG was digitized at a 64-bit resolution with a sampling rate of 512 Hz. This BioSemi system replaces the ground electrodes used in conventional systems with two separate electrodes: Common Mode Sense active electrode and Driven Right Leg passive electrode. These two electrodes form a feedback loop, which creates a zero-ground system (http://www.biosemi.com/faq/cms%26drl.htm). Data was recorded using ActiView software.

Data was preprocessed using CURRY 7 software [42]. Data was filtered offline with a 0.01–30 Hz bandpass. Waveforms fluctuating ± 200 μv within 100 ms were automatically marked bad and removed from the data. Data were baseline correct and a common average rereference (CAR) was applied to the data. Eye blinks were corrected using an average template generated from each individual participant. The template identified the VEOG channel as the artifact channel for eye blinks and performed a covariance analysis between this channel and each other EEG channel. Linear transmission coefficients were computed and based on the weights, a proportion of the voltage was subtracted from each data point in the eye blink interval. Finally, data were manually screened for any remaining artifacts via visual inspection of the EEG data.

#### Computer equipment

All instructions and tasks were completed on a Dell Precision T3500 Intel Xeon, Pentium class computer using E-Prime Professional v. 2.0.

#### Affective norms for English words

Word stimuli were obtained from the American Norms for English Words (ANEW) [43]. The ANEW is a set of English words that have been normed on a 9-point self-assessment manikin (SAM) for valence (1 = most unpleasant, 9 = most pleasant) and arousal (1 = most calming, 9 = most exciting). Thirty negative and thirty neutral words were selected. Negative and neutral words significantly differed on valence and arousal, but they did not significantly differ on average word length or frequency of use in the English language [44; see Table 1].

**Table 1:** Valence, arousal, word length, and frequency for negative and neutral words.

	Valence	Arousal	Word Length	Frequency
Negative	2.33 (0.29)	6.82 (0.44)	5.97 (1.43)	20.3 (30.08)
Neutral	4.84 (.41)	3.99 (.28)	6.10 (1.40)	39.67 (64.80)

The average normed score for negative and neutral words is shown with standard deviations in parenthesis.

#### Flanker stimuli

The Flanker task was adapted from Eriksen and Eriksen [40]. Flanker stimuli consisted of arrowheads and were presented congruently (>>>>> or <<<<<), incongruently (<<><< or >><>>), or neutrally (—>—or—<—). Targets are instructed to respond using only the central arrowhead, and to indicate whether the central arrowhead is facing left or right with a button press.

#### Self-report measures

*Spielberger State-Trait Anxiety Inventory (STAI)*. The STAI provides measures of the temporary condition of "state anxiety" and the more general and long-standing quality of "trait anxiety" in adults [45]. The STAI consists of two scales containing 20 items each. STAI Y-1 addresses state anxiety by evaluating how the subject feels "right now, at this moment", while the STAI Y-2 addresses trait anxiety by evaluating how the subject feels "generally". It uses “I feel/I am” statements that are rated on a 4-point scale from 1 (Not at All) to 4 (Very Much So). The STAI has an internal reliability coefficient alpha of .86-.95.

*Penn State Worry Questionnaire (PSWQ)*. The PSWQ is a measure of trait worry, or anxious apprehension [46]. It consists of 16 items rated on a 5-point Likert scale from “Not at all typical of me” to “Very typical of me”. The PSWQ has an internal reliability coefficient alpha of .93.

*Mood and Anxiety Symptom Questionnaire (MASQ)*. The MASQ is a measure of mood that contains subscales for anxious arousal and anhedonic depression [47]. It consists of 39 items rated on a 5-point Likert scale from “Not at all” to “Extremely” and has an internal reliability coefficient alpha of .78.

*Positive and Negative Affect Scale (PANAS) general*. The PANAS is a widely-used measure of trait mood state [48]. It includes a list of 20 adjective descriptors of 10 positive (e.g., “interested”, “enthusiastic”) and 10 negative (e.g., "irritable”, “upset”) affects. Items are rated on a 5-point scale from 1 (“very slightly or not at all”) to 5 (“extremely”) according to what extent [the person] feels this way in general. The positive affect subscale has an internal reliability coefficient alpha of .88, and the negative affect subscale has an internal reliability coefficient alpha of .87.

*Perceived Stress Scale (PSS)*. The PSS provides a measure of the degree to which one perceives life events as stressful [49]. The PSS consists of 14 items rated on a 5-point Likert scale from 0 (never) to 4 (very often). The PSS has an internal reliability coefficient alpha of .85.

*Self-Compassion Scale (SCS)*. The SCS [50] is a measure of self-compassion. It consists of 26 items rated on a 5-point Likert scale from “Almost Never” to “Almost Always”. Participants are asked to indicate how often they behave in various ways. The SCS has an internal reliability coefficient alpha of .92.

*Toronto Empathy Questionnaire (TEQ)*. The TEQ is a self-report measure of empathy created by Spreng and colleagues [51]. It contains 16 items rated on a 5 point Likert scale from “Never” to “Always”. The TEQ has an internal reliability coefficient alpha of .87.

### Procedure

Procedures for both pre- and post-training sessions were identical. Participants provided written, informed consent prior to providing any data for the study. At this point the study already obtained IRB approval. A demographic form was completed by each participant. Subsequently, the participants were set-up with the EEG equipment and seated in an electrically shielded, sound attenuated recording booth. In this booth, participants were read instructions on the task before completing a practice phase of the emotional Flanker task. The task timing was adapted from Larson and colleagues’ Flanker task [52]. The practice phase consisted of 10 trials followed by two blocks of experimental trials consisting of 90 trials each (180 trials total). Fifty-percent of trials had negative word stimuli and 50% had neutral word stimuli. Distribution of congruent, incongruent, and neutral flanker stimuli was equal across each word type, resulting in 30 trials of each trial type (negative-congruent, negative-incongruent, negative-neutral, neutral-congruent, neutral-incongruent, neutral-neutral). For each trial word stimuli were forward masked by a row of X’s (“XXXXXXXX”) that were presented for 150ms, followed by presentation of a word stimulus for 150 ms, followed by a backward mask identical to before for 150 ms. Forward and backward masking was used to disrupt elaborate processing of the word stimuli so that ERP responses to the words were not contaminating the ERP responses to the flanker stimuli. The flanking arrowheads of the flanker stimuli were then presented for 100 ms followed by the presentation of the center arrowhead for 2000 ms. Presentation of the flanker stimulus terminated upon response. A fixation sign (“+”) was presented during the intertrial interval, which randomly jittered between 1500–2000 ms. Participants responded using a keyboard pressing either the letter key ‘C’ or ‘M’ to indicate if the center arrowhead was facing left (C) or right (M). Presentation of word and flanker stimuli for each block was fully randomized between participants. A visualization of the Emotional Flanker Task can be found in Fig 2.

**Fig 2:** Timing of the emotional Flanker task. The arrow indicates the progression of time through a single trial of the Emotional Flanker Task.

Self-report measures were completed online via Qualtrics for both pre- and post-training assessments on the participants’ own time. Participants who opted to participate in the self-report measures completed the pre-training assessment during the first three weeks of the academic semester and the post-training assessment during the last three weeks of the semester. Order of self-report measure was fully randomized across participants and time. Class tests were completed during the regularly scheduled class periods and dates.

### Data processing

Our dependent variables were reaction time to the Flanker stimulus, ERP amplitudes in response to flanker stimuli, self-report measure scores, and test grades (out of 100). Reactions times and ERP amplitudes to correct trials only were analyzed. Our independent variables were Group (FA, SC), Time (pre-training, post-training), Valence (negative, neutral) and Congruency (congruent, incongruent, neutral). For the ERP data, epochs of 1000 ms after onset of Flanker stimuli were created, corrected to a 200 ms pre-stimulus baseline. Epochs for each trial type were then averaged together to produce ERPs. All participants had no more than 10 percent of trials removed. Subsequently, grand average waveforms were computed by averaging individual participant averages together. The grand averages were used to identify the ERP windows for the ERPs of interest. Typical windows for the N2 and P3 windows were extracted from each individual participant average before analyzing the midline channels to find the peak of each component. Previous research using affective primes in a Flanker task found the N2 to appear 320–380 ms post Flanker onset [35]. For this data, the N2 component was identified during the 300–360 ms window and was found to be largest at channel Fz. Channels Fz, F1, F2, AFz and CFz were averaged together to represent the scalp topography of the N2 component. Previous research examining the effects of stimulus valence on the P3 found the P3 to appear 300–600 ms post-stimulus onset [18]. For this data, the P3 component was identified during the 270–470 ms window and was found to be largest at channel POz. Channels POz, PO3, PO4, Pz, and Oz were averaged together to represent the scalp topography of the P3 component. These topographies are comparable to Atchley and colleagues [9].

## Results

### Self-report measures

Independent samples *t*-tests were conducted on pre-training survey scores between the Focused Attention and Self Compassion groups to ensure that no pre-existing differences between groups on these measures existed. No significant differences were found, all *p*’s > .05. For each self-report measure, 2 (Time: pre, post) by 2 (Group: FA, SC) mixed ANOVAs were then conducted, N = 44 (N = 43 for the PSWQ and STAI due to one participant not responding to all survey items). Significant interactions were broken down by calculating difference scores (post—pre) and conducting posthoc t-tests on the difference scores between the two groups. No significant main effects or interactions were found for the Toronto Empathy questionnaire, the Self-Compassion Survey, Negative Affect, and Anxious Arousal, all *p*’s > .05. A significant main effect of Time was found for the Penn State Worry Questionnaire, *F*(1, 41) = 6.16, *p* = .02, η_p_^2^ = .13, such that pre-training scores (*M* = 58.02, *SD* = 13.72) were higher than post-training scores (*M* = 54.91, *SD* = 14.39) overall. Both the main effect of Group and the interaction between Time and Group on PSWQ scores were not significant, *p*’s > .05.

A significant main effect of Time on Trait Anxiety was found, *F*(1, 41) = 8.00, *p* = .01, η_p_^2^ = .16, such that pre-training scores (*M* = 45.72, *SD* = 8.71) were higher than post-training scores (*M* = 42.81, *SD* = 9.01). A significant interaction between Time and Group was also found for Trait Anxiety scores, *F*(1, 41) = 5.36, *p* = .03, η_p_^2^ = .12. The difference score for Trait Anxiety was found to be significantly different between groups, *t*(41) = 2.32, *p* = .03, *d* = .70, *M*_*diff*_ = 5.26. Trait anxiety stayed relatively stable for the FA group (*M*_*diff_FA*_ = -0.58, *SD* = 6.67) but reduced following the training in the SC group (*M*_*diff_SC*_ = -5.84, *SD* = 8.23).

No significant main effects for Time or Group were found for Perceived Stress scores, however, a significant interaction was found, *F*(1, 42) = 7.17, *p* = .01, η_p_^2^ = .15. The difference score for Perceived Stress was found to be significantly different between groups, *t*(42) = 2.68, *p* = .01, *d* = .80, *M*_*diff*_ = 6.12. Perceived stress was higher for the FA group following the training (*M*_*diff_FA*_ = 1.42, *SD* = 6.24) but reduced in the SC group (*M*_*diff_SC*_ = -4.70, *SD* = 8.87).

No significant main effects of Time or Group were found for Positive Affect, however, a significant interaction was found, *F*(1, 42) = 4.39, *p* = .05, η_p_^2^ = .10. The difference score for Positive Affect was found to be significantly different between groups, *t*(42) = -2.10, *p* = .04, *d* = .63, *M*_*diff*_ = -4.23. Positive Affect was reduced in the FA group following the training (*M*_*diff_FA*_ = -3.38, *SD* = 6.64) but relatively stable in the SC group (*M*_*diff_SC*_ = 0.85, *SD* = 6.69).

Finally, no significant main effects of Time or Group were found for Anhedonic Depression, however, a significant interaction was found, *F*(1, 42) = 9.47, *p* = .004, η_p_^2^ = .18. The difference score for Anhedonic Depression was found to be significantly different between groups, *t*(42) = 3.08, *p* = .004, *d* = .92, *M*_*diff*_ = 9.98. Anhedonic Depression was higher in the FA group following the training (*M*_*diff_FA*_ = 4.08, *SD* = 9.09) but reduced in the SC group (*M*_*diff_SC*_ = -5.90, *SD* = 12.40). See Table 2 for all self-report measures means and standard deviations.

**Table 2:** Self-report data.

		*n*	TEQ *M*(*SD*)	STAI* *M*(*SD*)	SCS *M*(*SD*)	PSWQ *M(SD)*	PSS* *M(SD)*
FA	Pre	24	51.4 (6.68)	44.1 (9.07)	53.3 (7.12)	55.0 (14.09)	26.2 (7.62)
	Post	24	50.7 (9.05)	43.5 (8.46)	51.5 (7.19)	53.3 (14.34)	27.7 (8.52)
	Difference		-0.70	-0.60	-1.80	-1.70	1.50
SC	Pre	20	53.5 (5.08)^+^	47.8 (7.99)^+^	53.1 (7.29)	61.8 (12.58)^+^	29.2 (9.24)
	Post	20	53.4 (5.52)^+^	41.9 (9.81)^+^	51.9 (6.96)	56.9 (14.58)^+^	24.5 (8.68)
	Difference		-0.10	-5.90	-1.20	-4.90	-4.70
		n	PA* *M(SD)*	NA *M(SD)*	MASQ AD* *M(SD)*	MASQ AR *M(SD)*	
FA	Pre	24	35.0 (7.11)	21.2 (6.55)	28.8 (9.28)	56.5 (18.15)	
	Post	24	31.7 (7.39)	21.2 (6.55)	32.9 (9.90)	56.5 (13.95)	
	Difference		-3.30	0.00	4.1	0.00	
SC	Pre	20	34.3 (7.01)	25.1 (7.87)	32.4 (13.37)	59.2 (15.78)	
	Post	20	35.1 (5.91)	22.4 (7.67)	26.5 (7.23)	53.4 (13.24)	
	Difference		0.80	-2.70	-5.90	-5.80	

FA = Focused Attention Mindfulness; SC = Self-Compassion Mindfulness; TEQ = Toronto Empathy Questionnaire; STAI = Trait Anxiety; PSWQ = Penn State Worry Questionnaire; PSS = Perceived Stress Scale.

^+^Missing one participant’s TEQ, STAI, and PSWQ self-report data.

*Indicates significant differences between group difference scores.

FA = Focused Attention Mindfulness; SC = Self-Compassion Mindfulness; PA = Positive Affect; NA = Negative Affect; MASQ AD = Questionnaire for Anhedonic Depression; MASQ AR = Questionnaire for Anxious Arousal

### Classroom performance

A 4 (Test: 1, 2, 3, 4) by 2 (Group: FA, SC) mixed ANOVA was conducted for class test scores, N = 52. No significant main effect of Test or Group was found, however, a significant interaction was found, *F*(3, 150) = 2.94, *p* = .04, η_p_^2^ = .06. Posthoc independent samples *t*-tests were conducted between group scores on each test. Test 1 occurred prior to any training beginning in either group. No significant difference on Test 1 grades was found between groups, *t*(50) = -0.88, *p* = .39, *d* = .24, *M*_*diff*_ = -3.15. Grades on Test 2 were found to be significantly different between groups, *t*(50) = -2.01, *p* = .049, *d* = .56, *M*_*diff*_ = -7.68. Grades for the SC group (*M* = 83.16, *SD* = 13.13) were significantly higher than grades for the FA group (*M* = 75.48, *SD* = 14.28). Grades on Test 3 were found to be significantly different between groups, *t*(50) = -2.81, *p* = .007, *d* = .79, *M*_*diff*_ = -10.16. Grades for the SC group (*M* = 86.92, *SD* = 10.51) were significantly higher than grades for the FA group (*M* = 76.76, *SD* = 14.97). No significant difference on Test 4 grades was found between groups, *t*(50) = -0.72, *p* = .48, *d* = .20, *M*_*diff*_ = -3.70. See Table 3 for all test grade means and standard deviations.

**Table 3:** Test grades by group.

	n	Test 1 *M(SD)*	Test 2* *M(SD)*	Test 3* *M(SD)*	Test 4 *M(SD)*
FA	27	79.8 (11.81)	75.5 (14.28)	76.8 (14.97)	80.4 (12.95)
SC	25	83.0 (14.05)	83.2 (13.13)	86.9 (10.51)	82.9 (11.99)

FA = Focused Attention Mindfulness; SC = Self-Compassion Mindfulness.

*Indicates a significant difference between groups.

### Emotional Flanker task behavioral performance

Accuracy on the Emotional Flanker task was near ceiling (pre: *M* = .98, *SD* = .03, post: *M* = .97, *SD* = .02) and did not significantly differ between groups (pre FA: *M* = .98, *SD* =. 01, post FA: *M* = .98, *SD* = .01, pre SC: *M* = .97, *SD* = .03, post SC: *M* = .97, *SD* = .03). A 4-way mixed ANOVA was conducted on reaction time (RT) data with Time (pre, post), Valence (negative, neutral), and Congruency (congruent, incongruent, neutral) as within subjects factors and Group (FA, SC) as a between subjects factor, N = 31. A significant main effect of Time was found, *F*(1, 29) = 10.53, *p* = .003, η_p_^2^ = .27, such that pre-training RT was slower (*M* = 519.95, *SD* = 88.70) compared to post-training RT (*M* = 479.40, *SD* = 62.55). A significant main effect of Valence was found, *F*(1, 29) = 4.43, *p* = .04, η_p_^2^ = .13, such that Negative trials had faster RT (*M* = 498.02, *SD* = 67.51) compared to Neutral trials (*M* = 501.33, *SD* = 70.00). A significant main effect of Congruency was found, *F*(2, 29) = 140.17, *p* < .001, η_p_^2^ = .83, such that all conditions significantly differed from each other in bonferroni-corrected pairwise comparisons (Congruent: *M* = 452.98, *SD* = 68.37; Incongruent: *M* = 566.25, *SD* = 83.57; Neutral: *M* = 479.80, *SD* = 63.29). A significant interaction between Valence and Congruency was found, *F*(2, 29) = 4.69, *p* = .01, η_p_^2^ = .14, bonferroni-corrected posthoc paired *t*-tests revealed that RT on Incongruent trials significantly differed between Negative (*M* = 560.85, *SD* = 81.07) and Neutral (*M* = 571.64, *SD* = 87.45) valences, *t*(30) = -2.67, *p* = .01, *d* = 13, but no differences between valence were found for Congruent or Neutral flanker trials, all *p*’s > .016. No other 2-way interactions were found to be significant, all *p*’s > .05.

A significant 3-way interaction among Time, Congruency and Group was found, *F*(2, 58) = 4.18, *p* = .02, η_p_^2^ = .13. To break down this interaction, levels of Valence were averaged together for each level of Congruency, and then interference (incongruent—neutral) and facilitation (congruent—neutral) scores were calculated. Paired samples *t*-tests were then conducted on pre and post interference and facilitation scores for each group. For the FA group, post interference scores (*M* = 79.91 ms, *SD* = 38.24) were significantly reduced compared to pre interference scores (*M* = 108.82 ms, *SD* = 62.06), *t*(14) = 2.70, *p* = .02, *d* = .56, *M*_*diff*_ = 28.91 ms, and no significant difference on pre/post facilitation scores was found, *p* > .05. For the SC group, no significant pre/post differences were found on interference or facilitation scores, *p’s* > .05. The 4-way interaction was not found to be significant, *p* > .05.

### Exploratory ERP analyses

Post-testing sample size for ERPs were greatly impacted. Of note, only 11 individuals in each group returned and had usable EEG data for analysis. As such, the ERP analyses for the Emotional Flanker Task should be considered exploratory in nature, N = 22.

#### N2 ERP

The same 4-way mixed ANOVA was conducted on ERP amplitudes. A significant 2-way interaction between Valence and Congruency was found, *F*(2, 44) = 3.23, *p* < .05, η_p_^2^ = .13. A significant 3-way interaction among Time, Valence, and Congruency was found, *F*(2, 44) = 4.14, *p* = .02, η_p_^2^ = .16. These were qualified by a significant 4-way interaction among Time, Valence, Congruency and Group was found for the N2 amplitude, *F*(2, 44) = 5.79, *p* = .01, η_p_^2^ = .21. To break down this interaction, interference and facilitation effects were calculated the same way as was done for RT but without collapsing across levels of Valence. A significant 3-way interaction was found among Time, Valence, and Group, *F*(1, 20) = 11.44, *p* = .003, η_p_^2^ = .36. This was followed by paired samples *t*-tests for each Group. For the FA group, no significant N2 effects were found, all *p’s* > .05.

For the SC group, the N2 response on negative-valence trials was significantly reduced in the post data (*M* = -5.73 μv, *SD* = 4.64) compared to the pre data (*M* = -7.20 μv, *SD* = 5.37), *p* = .004. No significant differences were found between the pre and post neutral-valence trials, *p* > .05 (see Fig 3). All other main effects and interactions were not significant, *p’s* > .05.

**Fig 3:** Grand average waveforms showing the effect of group and time on negative prime trials on N2 amplitude at channel Fz. The solid lines indicate the grand average waveforms for the negative-valence Flanker trials pre-training. The dashed lines indicate the grand average waveforms for the negative-valence Flanker trials post-training.

#### P3 ERP

For the P3 amplitude, a significant main effect of Congruency was found, *F*(2, 44) = 4.57, *p* = .02, η_p_^2^ = .17, such that neutral trials elicited larger P300 responses (*M* = 6.06, *SD* = 3.62) compared to congruent trials (*M* = 4.47, *SD* = 3.61), but not incongruent trials (*M* = 4.70, *SD* = 3.50). A significant 4-way interaction among Time, Valence, Congruency and Group was found for the P3 amplitude, *F*(2, 44) = 6.04, *p* = .005, η_p_^2^ = .22. To break down this interaction, interference and facilitation effects were calculated the same way as for the N2 data. A significant 3-way interaction was found among Time, Valence, and Group, *F*(1, 20) = 13.24, *p* = .002, η_p_^2^ = .40. This was followed by paired samples *t*-tests for each Group. For the FA group, no significant P3 effects were found, all *p’s* > .05.

For the SC group, the P3 response on negative-valence trials was significantly reduced in the post data (*M* = 4.33 μv, *SD* = 2.77) compared to the pre data (*M* = 5.62 μv, *SD* = 3.78), *p* = .01. No significant differences were found between the pre and post neutral-valence trials, *p* > .05 (see Fig 4). All other main effects and interactions were not significant, *p’s* > .05.

**Fig 4:** Grand average waveforms showing the effect of group and time on negative prime trials on P3 amplitude at channel POz. The solid lines indicate the grand average waveforms for the negative-valence Flanker trials pre-training. The dashed lines indicate the grand average waveforms for the negative-valence Flanker trials post-training.

## Discussion

Our results indicate that different types of mindfulness practices do have unique effects on wellbeing and attentional control. We were able to support our hypothesis that FA practice would lead to better indices of attentional control, though this was only evident in the reaction time and not the ERP data. We were also able to support our hypothesis that SC practice would lead to better indices of wellbeing and attentional control in the presence of emotional distraction. This was evident in several of the self-report measures of wellbeing, as well as in reduced N2 and P3 ERP responses to flanker stimuli with negative primes. Further, the SC group was found to outperform the FA group on three of four class tests after the practices were incorporated into the classroom, supporting the hypothesis that the SC group would experience greater testperformance, however, our data indicate that this only occured on a short term basis.

Mindfulness practices have been associated with improved cognition, particularly attention, in neuroimaging and behavioral research [17–19, 53, 54]. As such, the FA group in this study having reduced interference effects on the Flanker task after training, regardless of emotional primes, supports this association. We were expecting this improvement in behavioral performance to be accompanied by neural indices of improved cognition, however, no differences in the ERP responses to the stimuli were found in the FA group. This may indicate that different mechanisms were being employed by the group to improve performance, so no one ERP component captured the cognitive effect. Similar research which employed the Stroop task to assess the impact of FA meditation on attentional control [39] saw no significant ERP effects after 8 weeks, but did find neural indices of improved attention after 16 weeks. The current study’s intervention lasted 10 weeks, so perhaps given more time, we too would have seen attention effects on the ERP components.

The SC group showed significant improvement in emotional regulation after training. On the Emotional Flanker task, individuals in the SC group had reduced N2 and P3 responses to stimuli with negative primes. This indicates that the negative words used to prime the flanker stimuli were being processed more efficiently and were causing less distraction for the SC group, regardless of the congruency of the Flanker stimulus. While these neural effects did not correspond with behavioral effects during the task in our study, this improved efficiency at processing emotional information may lead to individuals having more resources for other tasks in a more complex, real-life context. In other words, the changes in N2 and P3 amplitude in the SC group indicate improved attentional control. Further, while studying the effects of FA mindfulness, Moore and colleagues also had significant ERP effects without corresponding behavioral effects following 16 weeks of mindfulness training [39]. Another possible explanation for the reduced ERP response following negative words is that the SC group developed equanimity through their practices. Equanimity comes from the development of a non judgemental attitude toward stimuli, so that they are judged as neither good nor bad. While this construct is theorized to facilitate emotional regulation a reliable tool for assessing equanimity is still needed [for a review, see 55]. Equanimity could also explain why the SC group showed reduced neural responses following negative words that did not correspond with faster reaction times.

The ERP changes in the SC group do correspond with their self-reported wellbeing. The SC group showed significant reductions in trait anxiety, perceived stress, and anhedonic depression following the training. Again, this supports that the SC training is improving emotional regulation in this group. The FA group showed significant reductions in positive affect following the training. We do not think that this is a reflection of the FA practice causing reductions in mood, rather, we interpret this as the FA practice not helping build resiliency to the normal stresses of a college semester. The pre-training data was collected during the first three weeks of the semester, and the post-training data was collected during the last week and a half. It is normal for college students to experience lower mood states during the end of the semester when time management and workload pressures are higher [56].

The literature on the effects of mindfulness practices on education has been steadily growing for the past several decades. This is because of the consistent positive effects mindfulness practices have on the school behavior, wellbeing, and classroom performance of K-12 students [1, 2, 21] and college students [3]. Research studying these effects in post-secondary students is not as abundant; however, there is no reason to suspect that college-aged students cannot benefit from these practices as well. Indeed, the benefits of mindfulness practices for university students have been proposed [57] and found when investigated [20, 58], with the exception of one study that did not find behavioral benefits from mindfulness practice [59]. This study finds that even brief, 5 minute mindfulness practices incorporated into the start of a class can improve student wellbeing, attention, and test performance, particularly if the practice focuses on self-compassion. An intervention such as this is much more feasible for the average instructor to incorporate than more rigorous and time-consuming MBIs that have been studied.

We did not have a control group in this study, so it is possible that both the FA and SC groups’ classroom performance benefitted from these practices. Nonetheless, the SC group significantly outperformed the FA group on class tests after the training started. Again, we do not interpret this as the FA practice not having benefits on cognitive ability and classroom learning. Rather, we think this strongly supports the literature from K-12 education that indicates the importance of socioemotional wellbeing on learning and education [1, 2]. It is not surprising that students who were experiencing less anxiety, stress, and depression were performing better on class tests, as these negative mood states are associated with reductions in working memory, attentional control, and executive functioning [60]. Further, the SC group outperforming the FA group on class tests 2 and 3, but not test 4, is inline with a study that found mindfulness practices to benefit short-term academic performance but not long-term [20]. Because the two groups did not change in the same way on any of our measures, we do not think that these results are due to the passage of time or practice effects.

Putting all of our results together, different time-courses for cognitive and emotional effects of FA vs. SC mindfulness practices are suggested. The FA practice did not significantly impact neural indices of attention in the time course of our intervention. However, it is likely that given more practice, the behavioral improvements observed in the FA group can start to benefit attentional processing and more applied assessments of cognition, such as classroom tests. For example, Moore and colleagues found no behavioral or neural effects of breath-focused mindfulness at 8-weeks of intervention but did find ERP effects at 16 weeks of intervention [39]. Indeed, complex relationships among attentional control mechanisms and emotion regulation abilities have been established and widely studied [for a meta-analysis see 61].

In contrast, the SC practice seems to serve as a double-edged sword. Both attentional control and emotional regulation abilities seem to be simultaneously exercised in this practice. As such, larger benefits are seen neurally and in self-reports of wellbeing sooner in individuals who practice SC mindfulness. These gains in cognition and emotional regulation likely contribute to classroom performance by improving attention and reducing emotional distraction, such as anxiety, possibly landing students in the ideal zone for performance given a moderate level of physiological arousal [62]. Again, the relationship among these variables has been established in the literature [63].

### Limitations and future directions

Due to the applied nature of this study, sample sizes for different dependent variables vary based on the ease of student participation. As such, the final sample size for pre-/post-training ERP data is relatively small; however, we did obtain effect sizes for this data that fall within the range of effect sizes for the effects of mindfulness on physiology from a recent meta-meta analysis [7]. Nonetheless, further replications of these effects with larger sample sizes will be needed to determine their reliability.

It should also be noted that the lead author for this paper was also the instructor for the courses from which the participants were recruited. While not present during data collection in an effort to reduce demand characteristics, the students were aware that the research was being conducted by their professor. Due to the nature of conducting a class intervention students were not randomly selected into groups, instead the classes as a whole were randomly selected to a group. Furthermore, unlike most studies that use daily practice for the interventions, the FA and SC groups only received five minutes of practice twice a week. Finally, the two classes that were randomly assigned to the FA vs. SC training were identical except for the time of day at which they occurred. The FA group’s class was in the mid-morning, and the SC group’s class was in the early afternoon. Time of day, as well as class dynamics, may have differentially impacted the emotional states and test performance of the students. Replication studies that can control for these effects will help contribute to the reliability of these effects.

## Conclusions

Students who practice mindfulness as part of their college courses show cognitive and wellbeing benefits, depending on the type of mindfulness practice, even when only practicing for five minutes twice a week. Practicing focused-attention mindfulness, where attention is held on the sensation of the breath, had a minimal benefit in this study. Students showed indications of improved attentional control via reaction times to the incongruent flanker stimuli. This improvement in cognition did not appear to generalize to improvements in wellbeing or classroom performance following 10 weeks of practice. The benefits of self-compassion mindfulness, where attention is held on compassionate phrases toward the self, had broad benefits in this study. Students showed neural indications of improved attentional control when presented with negative information. This effect corresponded with multiple improvements in self-reported wellbeing and improved classroom performance in the short-term during the semester. Thus, if a singular practice were to be chosen for application in a small setting with relatively short practice, self-compassion mindfulness is indicated to be more beneficial.

## References

[1] ZennerC, Herrnleben-KurzS, WalachH. Mindfulness-based interventions in schools—a systematic review and meta-analysis. Front Psychol. 2014;5(603):1–20. doi: 10.3389/fpsyg.2014.00603 25071620PMC4075476

[2] ZoogmanS, GoldbergSB, HoytWT, MillerL. Mindfulness interventions with youth: a meta-analysis. Mindfulness. 2015;6(2):290–302. doi: 10.1007/s12671-013-0260-4

[3] ParsonsD, GardnerP, ParryS, SmartS. Mindfulness-based approaches for managing stress, anxiety and depression for health students in tertiary education: a scoping review. Mindfulness. 2022;13:1–16. doi: 10.1007/s12671-021-01740-3 34539929PMC8435111

[4] Kabat-ZinnJ. Mindfulness-based interventions in context: Past, present, and future. Clin Psychol: Sci Prac. 2003;10(2):144–156. doi: 10.1093/clipsy.bpg016

[5] BiedermannB, De LissaP, MahajanY, PolitoV, BadcockN, ConnorsMH, et al. Meditation and auditory attention: An ERP study of meditators and non-meditators. Int J Psychophysiol. 2016;109:63–70. doi: 10.1016/j.ijpsycho.2016.09.016 27693547

[6] ShapiroSL, CarlsonLE, AstinJA, FreedmanB. Mechanisms of mindfulness. J Clin Psychol. 2006;62(3):373–386. doi: 10.1002/jclp.20237 16385481

[7] GoldbergSB, RiordanKM, SunS, DavidsonRJ. The empirical status of mindfulness-based interventions: A systematic review of 44 meta-analyses of randomized controlled trials. Perspect Psychol Sci. 2021:1–23. doi: 10.1177/1745691620968771 33593124PMC8364929

[8] Kabat-ZinnJ, MassionAO, KristellerJ, PetersonLG, FletcherKE, PbertL, et al. Effectiveness of a meditation-based stress reduction program in the treatment of anxiety. Am J Psychiatry. 1992;149(7):936–943.160987510.1176/ajp.149.7.936

[9] AtchleyR, KleeD, MemmottT, GoodrichE, WahbehH, OkenB. Event-related potential correlates of mindfulness meditation competence. Neurosci. 2016;320:83–92. doi: 10.1016/j.neuroscience.2016.01.051 26850995PMC4777645

[10] Martin-AllanJ, LeesonP, LovegroveW. The effect of mindfulness and compassion meditation on state empathy and emotion. Mindfulness. 2021;12:1768–1778. doi: 10.1007/s12671-021-01639-z

[11] Pérez-ArandaA, García-CampayoJ, GudeF, LucianoJV, Feliu-SolerA, González-QuintelaA, et al. Impact of mindfulness and self-compassion on anxiety and depression: The mediating role of resilience. International Journal of Clinical and Health Psychology. 2021;21(2):1–9. doi: 10.1016/j.ijchp.2021.100229 33767736PMC7957152

[12] RocaP, VazquezC, DiezG, Brito-PonsG, McNallyRJ. Not all types of meditation are the same: Mediators of change in mindfulness and compassion meditation interventions. Journal of Affective Disorders. 2021;283:354–362. doi: 10.1016/j.jad.2021.01.070 33578349

[13] KlimeckiOM, LeibergS, RicardM, SingerT. Differential pattern of functional brain plasticity after compassion and empathy training. SCAN. 2014;9:873–879. doi: 10.1093/scan/nst060 23576808PMC4040103

[14] LippeltDP, HommelB, ColzatoLS. Focused attention, open monitoring and loving kindness meditation: effects on attention, conflict monitoring, and creativity–A review. Front Psychol. 2014;5:1083. doi: 10.3389/fpsyg.2014.01083 25295025PMC4171985

[15] GalanteJ, GalanteI, BekkersMJ, GallacherJ. Effect of kindness-based meditation on health and well-being: A systematic review and meta-analysis. J Consult Clin Psychol. 2014;82(6):1101. doi: 10.1037/a0037249 24979314

[16] HaukaasRB, GjerdeIB, VartingG, HallanHE, SolemS. A randomized controlled trial comparing the attention training technique and mindful self-compassion for students with symptoms of depression and anxiety. Front Psychol 2018;9:827. doi: 10.3389/fpsyg.2018.00827 29887823PMC5982936

[17] HildebrandtLK, McCallC, SingerT. Differential effects of attention-, compassion-, and socio-cognitively based mental practices on self-reports of mindfulness and compassion. Mindfulness. 2017;8:1488–1512. doi: 10.1007/s12671-017-0716-z 29201246PMC5693975

[18] ChiesaA, CalatiR, SerrettiA. Does mindfulness training improve cognitive abilities? A systematic review of neuropsychological findings. Clin Psychol Rev. 2011;31(3):449–464. doi: 10.1016/j.cpr.2010.11.003 21183265

[19] BrittonWB, DavisJH, LoucksEB, PetersonB, CullenBH, ReuterL, et al. Dismantling mindfulness-based cognitive therapy: Creation and validation of 8-week focused attention and open monitoring interventions within a 3-armed randomized controlled trial. Behav Res Ther. 2018;101;92–107. doi: 10.1016/j.brat.2017.09.010 29106898PMC5801080

[20] LinJW, MaiLJ. Impact of mindfulness meditation intervention on academic performance. Innov Educ and Teach Int. 2018;55(3):366–375. doi: 10.1080/14703297.2016.1231617

[21] FrancoC, MañasI, CangasAJ, GallegoJ. The applications of mindfulness with students of secondary school: Results on the academic performance, self-concept and anxiety. World Summit Knowl Soc. 2010:83–97. doi: 10.1007/978-3-642-16318-0_10

[22] BeaucheminJ, HutchinsTL, PattersonF. Mindfulness meditation may lessen anxiety, promote social skills, and improve academic performance among adolescents with learning disabilities. Complement Health Prac Rev. 2008;13(1);34–45. doi: 10.1177%2F1533210107311624

[23] LinY, FisherME, RobertsSMM, MoserJS. Deconstructing the emotion regulatory properties of mindfulness: An electrophysiological investigation. Front Hum Neurosci. 2016;10:1–13. doi: 10.3389/fnhum.2016.00451 27656139PMC5013076

[24] SangerKL, ThierryG, DorjeeD. Effects of school-based mindfulness training on emotion processing and well-being in adolescents: evidence from event-related potentials. Dev Sci. 2018;21(5):e12646. doi: 10.1111/desc.12646 29356254PMC6175003

[25] CahnRB, PolichJ. Meditation (vispanna) and the P3a event-related brain potential. Int J Psychophysiol. 2009;72:51–60. doi: 10.1016/j.ijpsycho.2008.03.013 18845193PMC2715145

[26] JoHG, SchmidtS, InackerE, MarkowiakM, HinterbergerT. Meditation and attention: A controlled study on long-term meditators in behavioral performance and event-related potentials of attentional control. Int J Psychophysiol. 2016;99:33–39. doi: 10.1016/j.ijpsycho.2015.11.016 26659014

[27] NorrisCJ, CreemD, HendlerR, KoberH. Brief mindfulness meditation improves attention in novices: Evidence from ERPs and moderation by neuroticism. Front Hum Neurosci. 2018;12:1–20. doi: 10.3389/fnhum.2018.00315 30127731PMC6088366

[28] Van der HurkPAM, GiommiF, CielenSC, SpeckensAEM, BarendregtHP. Greater efficiency in attentional processing related to mindfulness meditation. Q J Exp Psychol. 2010;63(6):1168–1180. doi: 10.1080/17470210903249365 20509209

[29] AndreuCI, CosmelliD, SlagterHA, FrankenIH. Effects of a brief mindfulness-meditation intervention on neural measures of response inhibition in cigarette smokers. PLoS ONE. 2018;13(1):e0191661. doi: 10.1371/journal.pone.0191661 29370256PMC5784955

[30] Dawson GC. The role of dispositional mindfulness in the development of emotion recognition ability and inhibitory control from late adolescence to early adulthood. 2020;[Doctoral dissertation, Case Western Reserve University]. OhioLink.

[31] DengX, ZhangJ, HuL, ZengH. Neurophysiological evidence of the transient effects of mindfulness induction on emotional processing in children: An ERP study. Int J Psychophysiol. 2019;143:36–43. doi: 10.1016/j.ijpsycho.2019.06.014 31269419

[32] IsbelBD, LagopoulosJ, HermensDF, SummersMJ. Mental training affects electrophysiological markers of attention resource allocation in healthy older adults. Neurosci Lett. 2019;698:186–191. doi: 10.1016/j.neulet.2019.01.029 30659914

[33] QuagliaJT, ZeidanF, GrossenbacherPG, FreemanSP, BraunSE, MartelliA, et al. Brief mindfulness training enhances cognitive control in socioemotional contexts: Behavioral and neural evidence. PLoS ONE. 2019;14(7):e0219862. doi: 10.1371/journal.pone.0219862 31323050PMC6641506

[34] KanskeP, KotzSA. Emotion triggers executive attention: ACC and amygdala responses to emotional words in a conflict task. Hum Brain Mapp. 2011;32(2):198–208. doi: 10.1002/hbm.21012 20715084PMC6870409

[35] DennisTA, ChenC-C. Trait anxiety and conflict monitoring following threat: An ERP study. Psychophysiol. 2009;46:122–131. doi: 10.1111/j.1469-8986.2008.00758.x 19055504PMC2701368

[36] LakeyCE, BerryDR, SellersEW. Manipulating attention via mindfulness induction improves P300-based brain-computer interface performance. J Neural Eng. 2011;8(2):025019. doi: 10.1088/1741-2560/8/2/025019 21436516PMC4429763

[37] PolichJ. Updating P300: An integrative theory of P3a and P3b. Clin Neurophysiol. 2007;118(10):2128–2148. doi: 10.1016/j.clinph.2007.04.019 17573239PMC2715154

[38] ConroyMA, PolichJ. Affective valence and P300 when stimulus arousal level is controlled. Cogn Emot. 2007;21(4):891–901. doi: 10.1080/02699930600926752

[39] MooreAW, GruberT, DeroseJ, MalinowskiP. Regular, brief mindfulness meditation practice improves electrophysiological markers of attentional control. Front Hum Neurosci. 2012;6:18. doi: 10.3389/fnhum.2012.00018 22363278PMC3277272

[40] EriksenBA, EriksenCW. Effects of noise letters upon the identification of a target letter in a nonsearch task. Percept Psychophys. 1974;16(1):143–149. doi: 10.3758/BF03203267

[41] JasperHH. The Ten-Twenty Electrode System of the International Federation. Electroencephalogr Clin Neurophysiol. 1958;10:371–375.10590970

[42] Compumedics Neuroscan. Curry 7 [Computer software]. 2008. compumedicsneuroscan.com/curry-7-signal-processing-basic-advanced-source-analysis/

[43] Bradley MM, Lang PJ. Affective norms for English words (ANEW): Stimuli, instruction manual and affective ratings. Technical report C-2, Gainesville, FL. The Center for Research in Psychophysiology, University of Florida.

[44] BrysbaertM, NewB. Moving beyond Kucera and Francis: A critical evaluation of current word frequency norms and the introduction of a new and improved word frequency measure for American English. Behav Res Methods. 2009;41(4):977–990. doi: 10.3758/BRM.41.4.977 19897807

[45] SpielbergerCD, GorsuchRL, LusheneRE. Manual for the State-Trait Anxiety Inventory. 1970. Palo Alto, California: Consulting Psychologists Press.

[46] MeyerTJ, MillerML, MetzgerRL, BorkovecTD. Development and validation of the Penn State Worry Questionnaire. Behav Res Ther. 199;28(6):487–495. doi: 10.1016/0005-7967(90)90135-6 2076086

[47] WatsonD, ClarkLA, WeberK, AssenheimerJS, StraussME, McCormickRA. Testing a tripartite model: I. evaluating the convergent and discriminant validity of anxiety and depression symptom scales. J Abnorm Psychol. 1995;104(1):3. doi: 10.1037//0021-843x.104.1.3 7897050

[48] WatsonD, ClarkLA, TellegenA. Development and validation of brief measures of positive and negative affect: the PANAS Scales. J Pers Soc Psychol. 1988;54(6):1063. doi: 10.1037//0022-3514.54.6.1063 3397865

[49] CohenS, KamarckT, MermelsteinR. A global measure of perceived stress. J Health Soc Behav. 1983:385–396. doi: 10.2307/2136404 6668417

[50] NeffKD. The development and validation of a scale to measure self-compassion. Self Identity. 2003;2(3):223–250. doi: 10.1080/15298860309027

[51] SprengRN, McKinnonMC, MarRA, LevineB. The Toronto Empathy Questionnaire: Scale development and initial validation of a factor-analytic solution to multiple empathy measures. J Pers Assess. 2009;91(1):62–71. doi: 10.1080/00223890802484381 19085285PMC2775495

[52] LarsonMJ, ClawsonA, ClaysonPE, BaldwinSA. Cognitive conflict adaptation in generalized anxiety disorder. Bio Psychol. 2013;94(2):408–418. doi: 10.1016/j.biopsycho.2013.08.006 24005064

[53] CahnRB, PolichJ. Meditation states and traits: EEG, ERP, and neuroimaging studies. Psychol Bull. 2006;132(2):180–211. doi: 10.1037/0033-2909.132.2.180 16536641

[54] Klopsis AL. The Impact of a Single Session of Mindfulness Meditation on the Attentional Blink in Non-Meditators. 2020;[Doctoral dissertation, CUNY]. CUNY Academic Works. academicworks.cuny.edu/gc_etds/3830

[55] WeberJ. A systematic literature review of equanimity in mindfulness based interventions. Pastoral Psychology. 2021;70:151–165. doi: 10.1007/s11089-021-00945-6

[56] MilyavskayaM, HarveyB, KoestnerR, PowersT, RosenbaumJ, IanakievaI, et al. Affect across the year: How perfectionism influences the pattern of university students’ affect across the calendar year. J Soc Clin Psychol. 2014;33(2):124–142. doi: 10.1521/jscp.2014.33.2.124

[57] BarbezatDP, BushM. Contemplative Practices in Higher Education. Jossey-Bass. 2014.

[58] Coo C, Escartin J. Less is more: the impact of mindfulness meditation on undergraduate students’ academic performance. Proceedings of INTED2018 Conference. 2018:9057–9059.

[59] WimmerL, DorjeeD. Toward determinants and effects of long-term mindfulness training in pre-adolescence: A cross-sectional study using event-related potentials. J Cogn Educ Psychol. 2020. doi: 10.1891/JCEP-D-19-00029

[60] CrockerLD, HellerW, WarrenSL, O’HareAJ, InfantolinoZP, MillerGA. Relationships among cognition, emotion, and motivation: implications for intervention and neuroplasticity in psychopathology. Front Hum Neurosci. 2013;7:261. doi: 10.3389/fnhum.2013.00261 23781184PMC3678097

[61] OchsnerKN, SilversJA, BuhleJT. Functional imaging studies of emotion regulation: a synthetic review and evolving model of the cognitive control of emotion. Ann N Y Acad Sci. 2012;1251:1–24. doi: 10.111.j.1749-6632.2012.06751.x2302535210.1111/j.1749-6632.2012.06751.xPMC4133790

[62] YerkesRM, DodsonJD. The relation of strength of stimulus to rapidity of habit-formation. J Comp Neurol Psychol. 1908;18(5):459–482.

[63] RoosAL, GoetzT, VoracekM, KrannichM, BiegM, JarrellA, et al. Test anxiety and physiological arousal: a systematic review and meta-analysis. Educ Psychol Rev. 2021;33:579–618. doi: 10.1007/s10648-020-09543-z

